The article "Computed Tomography Three-Dimensional Reconstruction Algorithm in the Diagnosis of Periodontitis and Its Correlation with Hypertension" was published in 2022. Journal: Comput Math Methods Med.

# Computed Tomography Three-Dimensional Reconstruction Algorithm in the Diagnosis of Periodontitis and Its Correlation with Hypertension

**DOI:** 10.1155/2022/1880178

**Published:** 2022-07-01

**Authors:** Lingling Xu, Jiaxin Pan, Jue Liu, Zhong Guan, Lu Zhao

**Affiliations:** ^1^Department of Stomatology, The Third Affiliated Hospital of Soochow University, Changzhou, Jiangsu 213003, China; ^2^Department of Gastrointestinal Surgery, The Third Affiliated Hospital of Soochow University, Changzhou, Jiangsu 213003, China

## Abstract

This study was aimed at exploring the value of iterative reconstruction (IR) algorithm to treat the periodontitis using computed tomography (CT) image and analyze the relationship between periodontitis and hypertension. 95 patients with periodontitis were selected, including 43 patients with periodontitis, 41 patients with advanced periodontitis and hypertension, and 11 patients with periodontitis and nonhigh blood pressure (NBP). The IR algorithm was introduced to the CT image scanning of them to reduce the noise. In addition, the CT value was statistically analyzed. High-sensitivity C-reactive protein (hs-CRP) and interleukin 6 (IL-6) were dramatically increased compared with periodontitis patients with NBP and with hypertension (*P* < 0.05). After the IR algorithm of the image, the quality, information, and mean square error (MSE) of the image were all effectively improved. Image with a 50% dose showed the lowest noise, but the reconstruction algorithm improved the low-contrast resolution. Moderate and severe periodontitis was independently related to hypertension. Inflammatory cytokines were independently related to hypertension of periodontitis patients (*P* < 0.05). Therefore, it was concluded that the IR algorithm could effectively improve the spatial resolution of the CT image when it was adopted to treat periodontitis and showed a high accuracy rate; the incidence of hypertension in patients with periodontitis was relatively high, and it had a certain relationship with periodontitis; and inflammatory cytokines were related to periodontitis and hypertension of patients.

## 1. Introduction

With the continuous improvement of people's lives and rapid economic development, people's lifestyles and dietary structure are also constantly changing. Chronic diseases such as hypertension, diabetes, and coronary heart disease (CHD) are also increasing frequently, and the relationship between hypertension and periodontitis has gradually become a research hotspot [1]. In severe cases, periodontitis will spread to the periodontal ligament, alveolar bone, cementum, and other deep periodontal tissues, which will cause chronic erosion of the alveolar bone and cause tooth loosening or falling off. Local inflammation in the periodontium will cause an increase in the level of C-reactive protein (CRP), so that vascular endothelial cells will be damaged [2]. The incidence of periodontitis in China as a whole is about 70%-85%. Periodontitis is a disease that endangers human oral health, and there is also a certain degree of correlation with the occurrence of hypertension [3]. Related studies have shown that periodontitis is related to the prevalence of hypertension, and the occurrence of hypertension will also cause the risk and severity of periodontitis. At this stage, the mechanism of action between the two is not particularly clear. The occurrence of inflammation is a mediator of the two diseases, and it is also a common risk factor, which can cause the disease to occur at the same time [4]. Hypertension and periodontitis are two relatively common diseases, and both have common risk factors, so it is particularly important to study the relationship between the two diseases [5]. IL-6 can cause endothelial dysfunction, increase peripheral vascular resistance, aggravate the occurrence of inflammatory factors, and ultimately cause damage to blood vessels.

The article "Computed Tomography Three-Dimensional Reconstruction Algorithm in the Diagnosis of Periodontitis and Its Correlation with Hypertension" was published in 2022. Journal: Comput Math Methods Med.

With the continuous use of computed tomography (CT) in clinical diagnosis, it is an important method for diagnosing periodontitis. The transmission effect formed by the destruction of the apical bone is the main basis for the clinical diagnosis of chronic periodontitis. In many cases, X-rays cannot provide enough information on the actual size of the lesion and the spatial location of the anatomical landmarks [6, 7]. CT has been extensively used in various fields. During CT scanning, the projection data on the detector is truncated due to different sizes of detector and object, and not all information of the object can be reflected by the reconstructed CT image. Therefore, it is necessary to reduce the clinical X-ray dose as much as possible, making the projection data incomplete, streak artifacts of the reconstructed image, and blurred detail information [8]. The range of the scanning angle becomes smaller due to some practical constraints in the industry. Under such a limited angle, there will be serious artifacts in reconstructed image. On the basis of the original equipment that does not affect the normal diagnosis, how to efficiently reduce the royal radiation dose to help the doctor in imaging has become a major issue in imaging [9]. Iterative reconstruction (IR) algorithm is a new infrared ray technology that can get the images conforming to the diagnostic requirements under lower scanning conditions. The calculation of IR algorithm is more, which takes a long time, and it is a good reconstruction method when the projection data were incomplete and with noisy [10]. The optimized CT reconstruction algorithm based on original CT collected data can reduce the noise on the image and improve the signal-to-noise ratio (SNR) of the image and thereby enhancing spatial and density resolution of the image. Therefore, it is of high significance to know the efficient reconstruction algorithms and apply them to the clinic [11]. Under the action of many factors, the bacteria in dental plaque and bacterial metabolites are the initiating factors of periodontitis, which will cause inflammation and affect the integrity of periodontitis.

The article "Computed Tomography Three-Dimensional Reconstruction Algorithm in the Diagnosis of Periodontitis and Its Correlation with Hypertension" was published in 2022. Journal: Comput Math Methods Med.

In this study, how to ensure the quality of reconstructed CT images was discussed. The most common methods for CT reconstruction were analytical reconstruction and statistical IR. Compared with the analytical reconstruction algorithm, the calculation of the IR algorithm was more flexible. The original image was reconstructed with projection data to obtain more accurate periodontitis treatment and diagnosis results, aiming to provide a reference for studying the correlation between periodontitis and hypertension.

## 2. Methods

### 2.1. General Data

Ninety-five patients with periodontitis who were hospitalized from March 2018 to January 2020 were selected to analyze the serum inflammatory cytokines, including 56 males and 39 females. They were aged 30-50 years old (41.24 ± 6.18 years old in average), 52 patients with hypertension and 43 patients with simple periodontitis. Patients meeting below criteria could be included: patients with no acute viral or bacterial infections, patients who were diagnosed as periodontitis after examination, and patients with no immune system diseases and no infectious diseases. Patients meeting the following criteria had to be excluded: patients with missed clinical data, patients who were forced to participate in this research, and patients with diseases in heart, liver, kidneys, hematopoietic system and diabetes. All patients had not received periodontal treatment in the past six months and had not used antibiotics within one month, except for complete dentition. This study had been approved by ethics committee of hospital. The family members of the patients gave informed consent to this study.

### 2.2. CT Scan

CT scan was performed as follows. Before the basic periodontal treatment, the patient should take a comfortable sitting position, the plane of the frame ears was parallel to the ground, and the head was placed in the CT scan frame to maintain the median dentition. After the CT scan, the data obtained was imported into the computer to reconstruct the data.

The article "Computed Tomography Three-Dimensional Reconstruction Algorithm in the Diagnosis of Periodontitis and Its Correlation with Hypertension" was published in 2022. Journal: Comput Math Methods Med.

The bleeding index of the teeth, plaque index, probing depth, and loss of attachment of patients were recorded. The diagnostic criteria for periodontitis were given as follows. It was determined as mild periodontitis if bleeding and inflammation were found in the gums, periodontal pocket was ≤4 mm, alveolar bone resorption was not over 1/3 of the root length, and attachment loss was 1-2 mm. It was determined as moderate periodontitis if attachment loss was 3-4 mm, teeth were slightly loosened, mild lesions were found in the root bifurcation area of multiple teeth, the gums suffered from inflammation, and there was pus. It was confirmed as severe periodontitis if there was obvious inflammation in the gums, periodontal was >6 mm, attachment loss was ≥5 mm, periodontal was abscess, there were bifurcation lesions for multiple roots, and teeth were loose.

Blood pressure was measured as follows. Before the measurement, the patient was required to relax, emptied the bladder, and keep calm and peace for 5 minutes. The patient sat on the seat with the backrest, bared the right upper arm, and kept the upper arm and blood pressure monitor were at the same level as the heart. The cuff covered at least 2/3 of the upper arm. The measurement should be repeated for twice to take the average value. If the systolic or diastolic blood pressure (SBP) or (DBP) was 5 mmHg between the two readings, it had to take another measurement and take the average of the 3 measurements. According to the 2010 Guidelines for the Prevention and Treatment of Hypertension in China, the grading criteria for hypertension with systolic blood pressure ≥ 140 mm, diastolic blood pressure ≥ 90 mmHg, history of hypertension, and taking antihypertensive drugs were determined as hypertensive patients. The reference range of normal blood pressure for Chinese adults was systolic blood pressure < 120 mmHg, and diastolic blood pressure < 80 mmHg.

### 2.3. Imaging Flow Chart of CT System

The imaging of CT images is similar to X-rays. X-rays pass through different tissues of the human body and have different gray levels on the CT images. After the X-rays penetrate, the corresponding attenuation levels of different tissues and organs are also different. CT images use highly collimated X-rays to scan a certain thickness of the patient's body. The detector records the attenuation information of the X-rays during the scanning process.  Figure 1 shows the imaging flow chart of the CT system. The converter converted analog information into digital information and then inputted it into electronic calculations. The information data stream passed through a high-voltage generator to provide power to generate X-rays. The CT machine also rotated at this time, and the detector continuously collected data and converted it into electrical signals according to the scan of the patient's body parts. Then, it was converted into digital electrical signals using the DAS system, and the image was reconstructed using the slip ring system.

The article "Computed Tomography Three-Dimensional Reconstruction Algorithm in the Diagnosis of Periodontitis and Its Correlation with Hypertension" was published in 2022. Journal: Comput Math Methods Med.

### 2.4. Improvement of Image Noise Using the IR Algorithm

The application process of iterative algorithm in CT image reconstruction is a process of model reconstruction. Firstly, a virtual image was constructed, and establishing an iterative model also included the construction of a noise model. According to the actual measurement value, the hypothetical image was continuously revised repeatedly to effectively control the noise level of each pixel to reach the desired level. The image of CT iteration consisted of two parts: front projection and back projection. The principle of SNR reduction is shown in Figure 2. The image assumptions and the initial value were set to obtain the projection value, and then, the image was repeatedly corrected. The SNR of the image was reduced to obtain the reconstructed image.

### 2.5. Principles of the Algorithm

The projection of a two-dimensional image with size of *A* × *A* is given in the equation below:

(1) $$\begin{array}{c} D=QH. \end{array}$$

In the equation above, *H* represented the image vector with size *AA* × 1; *Q* referred to the projection coefficient matrix (PCM) of *YW* × *AA*, *W* was the projection angle, *Y* was the maximum number of projections at each angle, and *D* referred to the projection vector with size *YW* × 1.

The reconstructed image was given as below:

(2) $$\begin{array}{c} B^{*}=Q^{*}D. \end{array}$$

In equation (2) above, *B*∗ was the reconstructed image with a size of *AA* × 1 and *Q*∗ represented the generalized inverse of the PCM *Q*. The direct calculation of *Q*∗ was complicated and consumed the time.

The first-order iterative method was used to obtain *Q*∗. If the initial estimate of generalized inverse *Q*∗ of the PCM *Q* of *YW* × *AA* was set to *N*_0_, and residual *S*_0_ = *D*_*R*(*T*)_ − *QN*_0_ was defined to meet *γS*_0_ < 1 (*γS*_0_ represented the spectral radius of *S*_0_, and *D*_*R*_(*Q*) was the orthogonal matrix of *Q*), then the sequence [*N*_0_, *N*_1_ ⋯ ⋯*N*_*K*_, *N*_*K*+1_, ⋯⋯] can be given in the following equation:

(3) $$\begin{array}{c} N_{K+1}=N_{k}+N_{0}-N_{0}{QN}_{K}\left(K=0,1\right)\cdots \cdots . \end{array}$$

When *K*⟶∞, *N* in equation (3) converged to *Q*∗; then, the sequence of the residual value met the following equation:

(4) $$\begin{array}{c} ║S_{K＋1}║\leq ║S_{0}║S_{K}║,K=0,1\cdots \cdots . \end{array}$$

The norm of any multiplication matrix conformed to *S*_*K*_ = *D*_*R*(*T*)_ − *QN*_*K*_.

The article "Computed Tomography Three-Dimensional Reconstruction Algorithm in the Diagnosis of Periodontitis and Its Correlation with Hypertension" was published in 2022. Journal: Comput Math Methods Med.

*N*_0_ of *Q*∗ was deemed to be equal to below equation:

(5) $$\begin{array}{c} N_{0}={qQ}^{t}. \end{array}$$

In equation (5) above, *Q*^*t*^ was the transposition of *Q*, and *θ* was an actual value, which conformed to the below equation:

(6) $$\begin{array}{c} 0<\theta <\frac{2}{\lambda 1\left({QQ}^{t}\right)}. \end{array}$$

In the equation above, *λ*_1_ (*QQ*^t^) referred to the largest nonzero eigenvalue of *QQ*^*t*^.

Two sides of equation (3) were multiplied by the *D* synchronously for easy calculation of *Q* and *Q*^*q*^, and the following equation could be obtained:

(7) $$\begin{array}{c} N_{K+1}D=N_{K}D+N_{0}D-N_{0}{QN}_{K}D,K=0,1\cdots \cdots . \end{array}$$

In the above equation, *N*_*K*+1_*D* and *N*_*K*_*D* represented the *K* + 1-th and *K*-th reconstructed images *H*^*i*^_*K*+1_ and *H*^*i*^_*K*_, respectively; *N*_0_*D* was the initial image *H*^*i*^_0_; *N*_0_*QN*_*K*_*D* referred to the projection of *H*^*i*^. In this study, the *θ* times of image reconstructed by filtered back projection (FBP) algorithm was used to replace the *N*_0_*QN*_*K*_*D*. When *AA* < *YW*, *θ* = 1; if *NN* > *YW*, *θ* < 2^−*AA*/*YW*^. Therefore, the above equation can be simplified as the following:

(8) $$\begin{array}{c} {H^{i}}_{K+1}={H^{i}}_{K}+{H^{i}}_{0}-N_{0}{{QH}^{i}}_{K}. \end{array}$$

The following experiments were carried out to verify the performance. The value of *θ* was 1 in this study.

The flow chart of IR algorithm is shown in Figure 3 below.

### 2.6. Steps of the Algorithm

Steps of the algorithm are shown in Figure 4. Firstly, *θ* and termination conditions *φ* were initialized. Secondly, when *K* = 0, the FBP algorithm reconstructed the image *H*^*i*^_fbp_ to obtain the preprocessed image *H*^*i*^_0_ = *θH*^*i*^_flp_. Thirdly, *H*^*i*^_*K*_ was projected to obtain the projection value *D*_*k*_. Fourthly, the image was reconstructed based on *D*_*k*_ according to FBP, and the result was multiplied by *θ* to get *H*_*r*_. Fifthly, image was corrected using the equation *H*^*i*^_*K*+1_ = *H*^*i*^_*K*_ + *H*^*i*^_0_ − *H*^*i*^_*r*_. Sixthly, Δ = ║*H*^*i*^_*K*+1−_ − *H*^*i*^_*K*_║≤*K* = *k* + 1 was defined. Finally, if Δ > *φ*, it had to return to step 3; otherwise, the operation was completed.

### 2.7. Observation Indicators

For the determination of inflammatory factors, 5 mL blood was collected on an empty stomach without anticoagulation, centrifuged at 3000 r/min for 10 minutes, and stored at -20°C. The latex-enhanced immunoturbidimetric method was used to determine the high-sensitivity C-reactive protein (hs-CRP). The interleukin-6 (IL-6) was determined by the double-antibody sandwich enzyme-linked immunosorbent assay (ELISA) method in the Roche automatic chemiluminescence analyzer. The determinations were performed in strict accordance with the instructions.

The article "Computed Tomography Three-Dimensional Reconstruction Algorithm in the Diagnosis of Periodontitis and Its Correlation with Hypertension" was published in 2022. Journal: Comput Math Methods Med.

### 2.8. Statistical Methods

All data were recorded using SPASS 21.0 to record relevant data of patients with chronic periodontitis. The measurement data were expressed in the form of *x̅*±sd and were analyzed using *T* test. The count data were displayed in the form of (*n*, %), and *P* < 0.05 indicated that there was a statistical difference. The analysis adopted multiple stepwise regression analysis.

## 3. Results

### 3.1. Comparison on General Data

Figure 5 shows a statistics of the general data of periodontitis patients. There were 23 male patients and 20 female patients with simple periodontitis, and the proportion of smoking patients was 39.76%. Periodontitis patients with hypertension included 27 males and 14 females, and the proportion of smokers was 42.16%. Among the periodontitis patients with NBP, there were 6 males and 5 females, and smoking patients accounted for 19.18%. Therefore, no statistical difference was found between patients in different groups (*P* > 0.05).

### 3.2. Preprocessed Images

Figure 6 shows the images with the same dose.  Figure 6(a) is the original image with low dose of a periodontitis patient, Figure 6(b) is the reconstructed image, Figure 6(c) shows the original image with low dose of the hypertension patient, and Figure 6(d) is the CT image of the patient after the reconstruction algorithm. The figure shows that the images reconstructed with FBP algorithm (Figures 6(a) and 6(c)) showed large noise and strong graininess. Figures 6(b) and 6(d) constructed using the IR algorithm show that the noise level and the smoothness of the image were improved greatly.

### 3.3. Reconstruction Results

Figure 7 shows a CT image of the alveolar bone of a patient. The patient came to the hospital with bleeding gums. After oral and other examinations, he was diagnosed with periodontal disease. The loose teeth were aggravated, and the gums were swollen. It can be seen from the CT image that the alveolar bone was resorbed obviously. Figures 7(a) and 7(b) show the lateral periodontal condition. The red circle in the figure marked the condition of the alveolar bone. Figures 7(c) and 7(d) show the condition of the alveolar bone in the upper and lower anterior teeth. The height of the alveolar bone was reduced, and the teeth were loose, displaced, and chewing weakness. Epidemiology showed that periodontal disease was the first reason for the loss of teeth in adults in China.

The article "Computed Tomography Three-Dimensional Reconstruction Algorithm in the Diagnosis of Periodontitis and Its Correlation with Hypertension" was published in 2022. Journal: Comput Math Methods Med.

### 3.4. Results of Reconstruction Algorithms

In Figure 8, noise of the image did not increase after using the iterative algorithm. With the decrease of the used dose, the spatial resolution of the image was effectively improved. As shown in Figure 9, the image with a 50% dose showed the lowest noise, but the reconstruction algorithm improved the low-contrast resolution.

### 3.5. MSE of CT Image Reconstructed with IR Algorithm

After iterations, the original image can be restored under IR algorithm (Figure 10). The closer the MSE is to zero, the better the effect. The figure revealed that the image quality was better after the reconstruction algorithm.

### 3.6. The Hypertension Inflammatory Cytokines of Periodontitis Patients

As illustrated in Figure 11, hs-CRP and IL-6 were dramatically increased in patients with NBP and hypertension compared with patients with periodontitis only (*P* < 0.05). However, periodontitis patients with hypertension showed no statistical significance compared with periodontitis patients with NBP (*P* > 0.05).

### 3.7. Multivariate Stepwise Regression Analysis

The hypertension was undertaken as the dependent variable, and the mild, moderate, and severe periodontitis were undertaken as the independent variables to perform a multivariate regression analysis, and it was found that moderate and severe periodontitis were independently correlated with hypertension (Figure 12). The relationship between inflammatory factors in serum and periodontitis was analyzed by taking inflammatory factors as independent variables and periodontitis as dependent variable. The results showed that inflammatory cytokines were independently related to the periodontitis with hypertension (Figure 13).

## 4. Discussion

Under the action of many factors, the bacteria in dental plaque and bacterial metabolites are the initiating factors of periodontitis, which will cause inflammation and affect the integrity of periodontitis. Periodontitis is a disease that endangers human oral health, and there is also a certain degree of correlation with the occurrence of hypertension. In severe cases, periodontitis will spread to the periodontal ligament, alveolar bone, cementum, and other deep periodontal tissues, which will cause chronic erosion of the alveolar bone and cause tooth loosening or falling off. Hypertension and periodontitis are two relatively common diseases, and both have common risk factors, so it is particularly important to study the relationship between the two diseases. Many epidemiological studies have been done on the relationship between periodontitis and hypertension. Statistics reported that the severity of periodontitis and systolic blood pressure showed a clear linear relationship among people aged 45-65. An average increase of 1.5 mmHg in systolic blood pressure will cause the degree of gum bleeding to increase by 10%, and the probability of diagnosis of hypertension will also increase by 1.1 times [12]. The results of Franek et al. [13] showed that periodontitis was related to the increase of central and systemic blood pressure, and the systolic blood pressure of primary hypertension increased with the severity of periodontitis. In this study, hypertension was undertaken as the dependent variable and the mild, moderate, and severe periodontitis were taken as the independent variables for multivariate regression analysis. It was found that moderate and severe were independently correlated with hypertension. Czesnikiewicz-Guzik et al. [14] studied the causal relationship between periodontitis and hypertension; inflammation is an important driving factor of hypertension, which was analyzed using a two-sample Mendelian randomization method; it proved that periodontitis-related single nucleotides were related to periodontitis GWAS and contraction, and the decrease in pressure was obviously correlated with the improvement of periodontal condition. Periodontitis is a chronic infectious disease caused by bacteria. The stimulation of inflammation increases the concentration of inflammatory transmitters in the blood. The increase of hs-CRP can damage vascular endothelial cells, affect the level of renin-angiotensin, and cause the occurrence of hypertension [15, 16]. IL-6 can cause endothelial dysfunction, increase peripheral vascular resistance, aggravate the occurrence of inflammatory factors, and ultimately cause damage to blood vessels [17, 18]. In this study, periodontitis patients with hypertension showed obviously higher hs-CRP and IL-6 levels compared with patients with periodontitis alone (*P* < 0.05).

The article "Computed Tomography Three-Dimensional Reconstruction Algorithm in the Diagnosis of Periodontitis and Its Correlation with Hypertension" was published in 2022. Journal: Comput Math Methods Med.

The application of reconstruction algorithms in CT images is not uncommon, and the algorithm can reduce image noise to a certain extent and improve the SNR. In this study, the reconstruction algorithm was applied to CT three-dimensional imaging. With the decrease of the used dose, the spatial resolution of the image was effectively improved. Comparison on the image noise suggested that the image with a 50% dose showed the lowest noise, but the reconstruction algorithm improved the low-contrast resolution. CT three-dimensional imaging increases the scanning speed and shortens the revolution time to 0.5 seconds, so it obtains multilayer images while rotating one revolution. The uninterrupted data collection can be performed on body fastly, obtaining more information [19]. After processing, some imaging techniques are completed, and the image quality is higher. The virtual endoscopy is not only more real but also improves the detection rate of smaller and mucosal lesions [20]. On this basis, IR algorithm reconstruction can effectively improve the image quality. The IR algorithm divides the entire image processing process into many times and gradually improves the image processing. In most low-dose scans, the image processing parameters of the scan have to be optimized to maximize the quality of the image. Algorithms and various noise reduction techniques can achieve the effect of smoothing the image [21]. In this study, the low-dose scans were adopted, and the results indicated that the IR algorithm showed good quality results in CT image scans of patients with periodontitis.

## 5. Conclusion

This work is aimed at exploring the value of IR algorithm in the treatment of periodontitis using CT images and to analyzing the relationship between periodontitis and hypertension. Quality of CT images was improved after optimization by IR algorithm, so that they were better with clear and intuitive visual field and simple steps, so the diagnosis effect of traditional CT in periodontitis was improved greatly. The conclusions of this study could be deemed as the foundation to analyze the periodontitis. There was a certain relationship between hypertension and periodontitis in patients with periodontitis, and there was a certain relationship between inflammatory cytokines and periodontitis and periodontitis with hypertension. The number of cases was not large, and the experiment can be combined with multiple centers at a certain time. The disadvantage of this work was that there were not many cases in the study, and the research object needed to be expanded. In addition, it was necessary to further explore low-dose CT imaging. Low-dose CT technology ensured image quality and could provide a diagnosis basis for treatment.

## Figures and Tables

**Figure 1:** Imaging flow chart of CT system.

**Figure 2:** Schematic diagram for improvement of image noise using IR algorithm.

**Figure 3:** The principle flow chart of IR algorithm.

**Figure 4:** Flow chart of algorithm.

**Figure 5:** General information of periodontitis patients.

**Figure 6:** Comparison on images under different algorithms with the same dose.

**Figure 7:** Three-dimensional CT image of severe periodontitis alveolar bone.

**Figure 8:** Quality evaluation on image using IR algorithm.

**Figure 9:** Improvement of signal-to-noise ratio (SNR).

**Figure 10:** MSE of images. A showed the MSE of CT image using IR algorithm; B showed the MSE of CT image without algorithm.

**Figure 11:** (a) The inflammatory cytokines of periodontitis patients. ∗ indicated that the difference was significant, *P* < 0.05. (b) The inflammatory cytokines in periodontitis patients with hypertension.

The article "Computed Tomography Three-Dimensional Reconstruction Algorithm in the Diagnosis of Periodontitis and Its Correlation with Hypertension" was published in 2022. Journal: Comput Math Methods Med.

**Figure 12:** Multivariate regression analysis results of periodontitis affecting hypertension. *β* and *P* represented two different correlation coefficients.

**Figure 13:** Multivariate regression analysis results of inflammatory factors affecting periodontitis with hypertension. *β* and *P* represented two different correlation coefficients.

## Data Availability

The data used to support the findings of this study are available from the corresponding author upon request.
